# Association between selenium intake and the risk of pancreatic cancer: a meta-analysis of observational studies

**DOI:** 10.1042/BSR20160345

**Published:** 2016-10-14

**Authors:** Lei Wang, Jianfeng Wang, Xudong Liu, Qian Liu, Guozhuan Zhang, Lishuang Liang

**Affiliations:** * Department of pain, Qilu Hospital of Shandong University, Ji'nan, Shandong 250000, P.R. China

**Keywords:** meta-analysis, pancreatic cancer, selenium

## Abstract

Quantification of the association between the intake of selenium and risk of pancreatic cancer is still conflicting. Thus, we conducted a meta-analysis to summarize the evidence from epidemiological studies of selenium intake with the risk of pancreatic cancer. Pertinent studies were identified by a search of PubMed and Web of Knowledge to July 2016. The random-effect model was used. Sensitivity analysis and publication bias were conducted. Data from six studies including 1424 pancreatic cancer cases were used in this meta-analysis. Pooled results suggested that highest selenium intake amount compared with lowest amount was significantly associated with the risk of pancreatic cancer [summary relative risk (RR)=0.659, 95% confidence interval (CI)=0.489–0.889, *I*^2^=47.6%]. The associations were significant both in case–control studies [RR=0.618, 95%CI=0.399–0.956, *I*^2^=59.1%] and Americas [RR=0.570, 95%CI=0.357–0.909, *I*^2^=65.6%]. No publication bias was found. Our analysis suggested that the higher intake of selenium might reduce the risk of pancreatic cancer.

## INTRODUCTION

Worldwide, pancreatic cancer causes more than a quarter of a million deaths annually and pancreatic cancer is the eighth commonest cause of death from cancer [1]. Generally, pancreatic cancer is most often diagnosed at a late stage. So, prognosis of pancreatic cancer is extremely poor with 1-year survival rates of 25% and 5-year survival rates of 4% [2,3]. However, because of the rarity of disease, general population would not choose the screening for pancreatic cancer. Therefore, it is very important to focus on risk or protective factors identification as a prevention strategy for pancreatic cancer. As we all know, several risk factors have been consistently associated with the risk of developing pancreatic cancer, including family history [4], chronic pancreatitis [5], cigarette smoking [6], diabetes mellitus [7] and obesity [8]. So, the protection factors for pancreatic cancer will be focused on the present study.

Selenium is a antioxidant mineral. It mainly presents in seafood, animal liver, kidney, egg products, nuts and other food. Selenium has been proposed to have many potential modes of action, including reducing oxidative DNA damage and genetic mutation [9,10]. Its composition suggested the protective potential for pancreatic cancer. For selenium intake and pancreatic cancer risk, the evidence from both case–control and cohort studies remains inconclusive. Therefore, we conducted a meta-analysis to assess the pancreatic cancer risk for the highest compared with lowest categories of selenium intake.

## MATERIALS AND METHODS

### Search strategy

Studies were identified using a literature search of PubMed and Web of Knowledge through July 2016 and by hand-searching the reference lists of the retrieved articles. The following search terms were used: ‘pancreatic cancer’ or ‘pancreatic carcinoma’ combined with ‘nutrition,’ or ‘diet,’ or ‘food,’ or ‘lifestyle,’ or ‘selenium’. Two investigators (LW and JFW) searched articles and reviewed all the retrieved studies independently. Disagreements between the two investigators were resolved by consensus with a third reviewer (XDL).

### Study selection

For inclusion, studies had to fulfil the following criteria: (1) have a prospective or case–control study design; (2) selenium intake was the independent variable of interest; (3) the dependent variable of interest was the incidence of pancreatic cancer; (4) relative risk (RR) or odds ratio (OR) with a 95% confidence interval (CI) was provided (or data available to calculate them). If data were replicated in more than one study, we included the study with the largest number of cases. Accordingly, the following exclusion criteria were also used: (1) reviews or letters; (2) repeated or overlapped publications; (3) those not report RR or OR; (4) animal studies.

### Data extraction

Two researchers (LW and JFW) independently extracted the following data from each study that met the criteria for inclusion: the last name of the first author, publication year, geographic locations, study design, the age range of study participants, duration of follow-up, the number of cases and participants and RR or OR (95%CI) for selenium intake and pancreatic cancer risk. From each study, we extracted the RR that reflected the greatest degree of control for potential confounders. If there was disagreement between the two investigators about eligibility of the data, it was resolved by consensus with a third reviewer (XDL).

### Statistical analysis

The pooled measure was calculated as the inverse variance-weighted mean of the logarithm of RR with 95% CI, to assess the association between selenium intake and pancreatic cancer risk. Random-effect model was used to combine study-specific RR (95%CI), which considers both within-study and between-study variation [11]. The *I*^2^ was used to assess heterogeneity, and *I*^2^ values of 0, 25, 50 and 75% represent no, low, moderate and high heterogeneity [12] respectively. Meta-regression with restricted maximum likelihood estimation was performed to assess the potentially important covariates that might exert substantial impact on between-study heterogeneity [13]. Publication bias was evaluated using Egger regression asymmetry test [14]. A study of influence analysis [15] was conducted to describe how robust the pooled estimator was to removal of individual studies. An individual study was suspected of excessive influence if the point estimate of its omitted analysis lay outside the 95% CI of the combined analysis. All statistical analyses were conducted with STATA version 11.0 (StataCorp LP). Two-tailed *P*-value ≤ 0.05 was accepted as statistically significant.

## RESULTS

### Search results and study characteristics

The search strategy identified 178 articles from PubMed and 203 from the Web of Knowledge, and 22 articles were reviewed in full after reviewing the title/abstract. Six articles [16–21] (three cohort studies and three case–control studies) involving 1424 pancreatic cancer cases were used in this meta-analysis after reviewed in full articles. The detailed steps of our literature search are shown in Figure 1. Three studies come from Americas, two from Europe, one from Australia. The characteristics of these studies are presented in Table 1.

**Figure 1:** The flow diagram of screened, excluded and analysed publications

**Table 1:** Characteristics of studies on selenium intake and pancreatic cancer risk

Study, year	Country	Study design	Participants (cases)	Age (years)	RR (95%CI) for highest compared with lowest category	Adjustment for covariates
Baghurst et al. (1991)	Australia	Case–control	357 (104)	<50 to ≥80	0.46 (0.23–0.94)	Adjust for age; pack-years of smoking, tobacco consumption and vice versa
Stolzenberg-Solomon et al. (2002)	Finland	Prospective	27111 (163)	50–69	0.91 (0.52–1.59)	Adjust for by the residual method and for age and years of smoking, energy-adjusted folate intake and energy-adjusted saturated fat intake
Gong et al. (2010)	United States	Case–control	2226 (525)	21–85	0.71 (0.54–0.95)	Adjusted for age in 5-year groups, sex and total energy intake, race, education, body mass index, history of diabetes, smoking, physical activity and alcohol consumption
Banim et al. (2013)	UK	Prospective	23658 (86)	40–74	0.79 (0.38–1.1)	Adjusted for age, sex, smoking, diabetes, total energy intake and body mass index category.
Han et al. (2013)	United States	Prospective	77446 (162)	50–76	0.79 (0.54–1.15)	Adjusted for age, gender, ethnicity, education, body mass index, physical activity, cigarette smoking status, total alcohol consumption, family history of pancreatic cancer, history of diabetes and total energy intake
Jansen et al. (2013)	United States	Case–control	1367 (384)	31–92	0.51 (0.34–0.76)	Adjusted for energy, smoking, BMI, age, sex and drinks of alcohol per week

### High compared with low analyses

Data from six studies including 1424 pancreatic cancer cases were used in this meta-analysis. Only two studies reported that selenium intake could reduce the risk of pancreatic cancer, whereas no significant association was reported in four studies. Pooled results suggested that highest selenium intake amount compared with lowest amount was significantly associated with the risk of pancreatic cancer [summary RR=0.659, 95%CI=0.489–0.889, *I*^2^=47.6%] (Figure 2).

**Figure 2:** The forest plot between highest compared with lowest categories of selenium intake and pancreatic cancer risk

In stratified analysis by study design, the associations was also found significant in the case–control studies [summary RR=0.618, 95%CI=0.399–0.956, *I*^2^=59.1%], but not in the prospective studies [summary RR=0.709, 95%CI=0.435–1.155, *I*^2^=49.6%]. In subgroup analyses for geographic locations, highest selenium intake level compared with lowest level was significantly associated with the risk of pancreatic cancer in Americas [summary RR=0.570, 95%CI=0.357–0.909, *I*^2^=65.6%], but not in Europe [summary RR=0.899, 95%CI=0.607–1.331, *I*^2^=0.0%]. The detailed results are summarized in Table 2.

**Table 2:** Summary risk estimates of the association between selenium intake and pancreatic cancer risk

				Heterogeneity test	
Subgroups	No. (cases)	No. studies	Risk estimate (95% CI)	*I*^2^ (%)	*P*-value
All studies	1424	6	0.659 (0.489–0.889)	47.6	0.089
Study design					
Case–control	1013	3	0.618 (0.399–0.956)	59.1	0.087
Prospective	411	3	0.709 (0.435–1.155)	49.6	0.138
Geographic locations					
America	1071	3	0.570 (0.357–0.909)	65.6	0.055
Europe	249	2	0.899 (0.607–1.331)	0.0	0.443

### Sources of heterogeneity and meta-regression

As seen in the pooled results, moderate heterogeneity was found in the analysis. In order to explore the source of between-study heterogeneity, univariate meta-regression was conducted. However, no significant findings were found in covariates of publication year (*P*=0.536), location where the study was conducted (*P*=0.792), study design (*P*=0.695) and number of cases (*P*=0.926).

### Influence analysis and publication bias

Influence analysis showed that no individual study had excessive influence on the association of selenium intake and pancreatic cancer risk (Figure 3). Egger's test (*P*=0.766) showed no evidence of significant publication bias between selenium intake and pancreatic cancer risk.

**Figure 3:** The influence analysis of selenium intake and pancreatic cancer risk

## DISCUSSION

Finding from this meta-analysis suggested that the higher intake of selenium might be able to reduce the risk of pancreatic cancer. The associations were also found in subgroups of case–control and Americas for selenium intake and pancreatic cancer risk.

Selenium is a trace element essential to human health. It plays an important role in thyroid hormone metabolism, antioxidant defense systems and immune function [22]. Selenium has several anti-carcinogenic mechanisms including inactivating oxygen free radicals, initiating DNA repair and inducing apoptosis [23]. Several epidemiological studies have indicated an inverse association between selenium intake and the risk of some cancers, such as prostate cancer [24], bladder cancer [25] and lung cancer [26], although the results were not all consistent [27]. In recent years, many studies had been performed to evaluate the relationship between selenium level and pancreatic cancer based on populations; however, the results were still conflicting. So, a hypothesis was conducted suggesting that higher intake of selenium might reduce the risk of pancreatic cancer. This hypothesis was verified by the results of this meta-analysis.

In this meta-analysis, moderate between-study heterogeneity was found in the pooled analysis and subgroup analysis. Although most studies in this meta-analysis used multivariate regression to adjust confounders, other indeterminate characteristics that varied among studies, such as publication year, location where the study was conducted, study design and number of cases etc. could be the causes of between-study heterogeneity. Hence, we used meta-regression to explore the potentially important covariate which could cause between-study heterogeneity. However, no aforementioned covariates had a significant impact on between-study heterogeneity. Pancreatic cancer is a complex aetiology and pathophysiology disease generated by the combined effects of genes and environment factors. Thus, other genetic and environment variables, as well as their possible interaction, may well be potential contributors to the heterogeneity observed.

As a meta-analysis of published studies, our findings showed some advantages. First, this is the first comprehensive meta-analysis of selenium intake and pancreatic cancer risk. Second, large number of cases and participants was included, allowing a much greater possibility of reaching reasonable conclusions between selenium intake and pancreatic cancer risk. Third, no significant publication bias was found, indicating that our results are stable.

However, there were some limitations in this meta-analysis. First, the associations were non-significant in prospective studies. These might because of only three studies with only 411 cases included in this meta-analysis. More studies with prospective design are wanted in the future studies. Second, measurement errors might exist in the assessment of dietary intake. This could lead to overestimation or underestimate the selenium intake magnitude [28,29]. Third, for the subgroups of geographic locations, the associations were only found significant in the Americas. Two studies with only 249 cases were conducted in Europe and only one study come from Australia. Due to this limitation, the results are applicable to the Americas, but cannot be extended to populations elsewhere. More studies originating in other countries are required.

In summary, results from this meta-analysis suggested that the higher intake of selenium might reduce the risk of pancreatic cancer.

## Abbreviations

CI: confidence interval
RR: relative risk
